The article "Clinical Study of Progesterone Combined with Vitamin B6 in the Treatment of Amenorrhea Endocrine Disorders Caused by Antipsychotics" was retracted in 2023. Reasons: signs of a paper mill; compromised peer review; unreliable results or conclusions.

# Clinical Study of Progesterone Combined with Vitamin B6 in the Treatment of Amenorrhea Endocrine Disorders Caused by Antipsychotics

**DOI:** 10.1155/2022/2436322

**Published:** 2022-08-28

**Authors:** Yijing Zhao, Shuangling Hu, Wenhui Zhai, Meijiao Wang, Lin Ran

**Affiliations:** ^1^Wuhan Wudong Hospital (Wuhan Second Psychiatric Hospital), 430084, China; ^2^Department of Obstetrics and Gynecology, Central Hospital of Enshi Tujia and Miao Autonomous Prefecture, 445000, China

## Abstract

**Background:**

Endocrine disorders such as amenorrhea, lactation, and irregular menstruation caused by antipsychotics are common in female patients. How to reduce or eliminate these adverse reactions is a matter of concern.

**Objective:**

To evaluate the therapeutic effect of progesterone in combination with vitamin B6 in the treatment of antipsychotic-induced amenorrhea.

**Methods:**

In our hospital, from May 2019 to May 2021, 120 patients with amenorrhea caused by antipsychotics who underwent surgery were selected for this prospective study. The random residue grouping method divided them into a progesterone group (60 cases) and a vitamin B6 group (60 cases). Among them, the progesterone group was treated only with progesterone, while the vitamin B6 group was given progesterone in combination with vitamin B6. The differences in endocrine index, prolactin, uterine size, and endometrial thickness, effectiveness, and safety analysis of the progesterone and vitamin B6 groups of patients were observed and compared.

**Results:**

Before treatment, there was no change in the comparison of endocrine indexes between the progesterone and vitamin B6 groups (*P* > 0.05). After 1 month of treatment, there were significant differences in estradiol, prolactin, and follicle-stimulating hormone between the progesterone and vitamin B6 groups of patients (*P* < 0.05). After 1 month of treatment, there were significant differences in prolactin, uterine size, and endometrial thickness, and the vitamin B6 group was significantly lower than the progesterone group (*P* < 0.05). The clinical efficiency of 95.00% in the vitamin B6 group was significantly higher than 83.33% in the progesterone group (*P* < 0.05). There were no adverse reactions in the progesterone and vitamin B6 groups.

**Conclusion:**

The effectiveness of progesterone combined with vitamin B6 in treating amenorrhea caused by antipsychotics is significantly better than simple progesterone, which can effectively improve the endocrine condition of patients and provide a reference for the clinical treatment of amenorrhea caused by antipsychotics.

## 1. Introduction

The occurrence of amenorrhea after taking antipsychotic drugs in female patients with psychosis is quite common. The incidence is as high as 17% to 78%, which directly affects the compliance of female patients to treatment and causes patients to discontinue treatment [1, 2]. Modern medical research has proved antipsychotics can cause abnormal metabolism and endocrine function, whether typical or atypical antipsychotics can cause blood prolactin to rise, leading to amenorrhea [3]. The mechanism is that antipsychotics block the dopamine D2 receptor on the prolactin cell membrane of the hypothalamus, reducing dopamine release. The prolactin secretion inhibitor decreases so that the secretion of prolactin increases, leading to amenorrhea in female patients. In addition, antipsychotics also inhibit luteinizing hormone and follicle-stimulating hormone, causing amenorrhea [4, 5]. It is difficult to recover after the occurrence of amenorrhea, which has different degrees of influence on the compliance of emotional medication in psychopaths, resulting in sexual dysfunction and a significant decrease in quality of life, thus affecting the rehabilitation of mental illness [6]. Psychiatric drugs promote a sharp increase in the secretion of prolactin in patients, which in turn leads to changes in the menstrual cycle of patients. Most patients have different degrees of irregular menstruation. In severe cases, they may even cause amenorrhea after medication. Progesterone and vitamin B6 combination therapy can reduce the patient's prolactin level and regulate the patient's menstrual cycle [7, 8]. Our study aims to explore the effectiveness and safety of vitamin B6 combined with progesterone in treating amenorrhea caused by antipsychotics. The current research results are reported as follows.

## 2. Materials and Methods

### 2.1. General Information

From May 2019 to May 2021 in our hospital, one hundred and twenty amenorrhea patients caused by antipsychotics who underwent surgery were selected. They were divided into a progesterone group and a vitamin B6 group (60 cases each) by the random residue grouping method. The progesterone group was treated only with progesterone, while the vitamin B6 group was given progesterone in combination with vitamin B6. Before the start of the study, patients and their families were informed to sign an informed consent by the principles of voluntariness, confidentiality, benefit, and harmlessness and have been approved by the medical ethics committee of our hospital. Patients with amenorrhea caused by antipsychotics meet the Chinese Classification and Diagnostic Criteria for Mental Disorders (CCMD-3) diagnostic criteria [9], excluding gynecological diseases and other physical diseases that can lead to amenorrhea and take risperidone or chlorpromazine for treatment. The therapeutic dose range of risperidone is 4-6 mg per day, and the therapeutic dose range of chlorpromazine is 400-650 mg per day. The duration of medication is more than one month. The menstruation before treatment is normal, and the amenorrhea is 3-6 months during the treatment. General data of the progesterone and vitamin B6 groups of patients had change in this test, as shown in Figure 1.

### 2.2. Inclusion and Exclusion Criteria

Inclusion criteria were menopause for more than 3 months after taking antipsychotic drugs, and patients with pregnancy and pregnancy-related diseases were excluded.

### 2.3. Method

The progesterone group was treated with progesterone monotherapy. Patients were given progesterone injection (manufacturer: Zhejiang Xianju Pharmaceutical Co., Ltd., approval number: National Medicine Zhunzi H33020828), intramuscular injection once a day, 20 mg each time. The vitamin B6 group was given a combined treatment of progesterone and vitamin B for 5 days (manufacturer: Zhejiang Ruixin Pharmaceutical Co., Ltd., approval number: National Medicine Zhunzi H33021137). Vitamin B6 tablets take orally 3 times a day, 80 mg each time, for 1 month. The above progesterone and vitamin B6 groups were treated with antipsychotic drugs according to the actual condition of the patients.

### 2.4. Follow-Up and Observation Indicators

(1) Endocrine indicators: Detect endocrine-related indicators of patients before treatment and 1 month after treatment, including prolactin, follicle-stimulating hormone, and estradiol. (2) The clinical treatment effect of amenorrhea patients is divided into cure: The symptoms and signs disappear; the marked effect is that the menstrual cycle of the patient is restored after treatment, and the patient's prolactin, follicle-stimulating hormone, and estradiol indicators return to normal; and the effect is that the patient's endocrine indicators have improved. The menstrual cycle is basically normal; invalid means that the patient's endocrine indicators have not improved, and menstruation is still irregular or continuous amenorrhea. Total effective = (cured + markedly effective + effective)/100.

### 2.5. Statistical Methods

Shapiro-Wilk method tested included data. Mean ± standard deviation ($\bar{x}$±S) described measurement data conforming to the normal distribution. The independent sample or paired-sample *t* test was implemented within the group, and the count data were described in whole numbers or percentages (%). Comparisons between groups or within groups were performed using the *χ*2 test. The data contained do not conform to the normal distribution and are described by M(QR) using the Mann-Whitney test, which has a test level of *α* = 0.05.

## 3. Results

### 3.1. General Information

The average age, amenorrhea time, taking antipsychotic drugs time, marital status, and other general data of the progesterone and vitamin B6 groups of patients were not different by *t*-test and chi-square test (*P* > 0.05) (see Table 1).

### 3.2. Comparison of Endocrine Indicators

Before treatment, there was no difference in the comparison of endocrine indexes between the progesterone and vitamin B6 groups (*P* > 0.05). After 1 month of treatment, there were significant differences in estradiol, prolactin, and follicle-stimulating hormone between the progesterone and vitamin B6 groups (*P* < 0.05) (see Table 2).

### 3.3. Comparison of Prolactin, Uterine Size, and Endometrial Thickness

After 1 month of prolactin treatment, the maximum diameter of the uterus, endometrial thickness, and prolactin of the vitamin B6 group was lower than the progesterone group (*P* < 0.05) (see Table 3).

### 3.4. Comparison of Clinical Efficacy and Poor Prognosis

The clinical treatment efficiency of the vitamin B6 group was 95.00%, which was significantly higher than that of the progesterone group (83.33%) (*P* < 0.05) (see Table 4).

## 4. Discussion

Among the commonly used antipsychotic drugs, either typical antipsychotic drugs or atypical antipsychotic drugs can cause amenorrhea. Its pathological mechanism includes two aspects. One is that antipsychotic drugs act on the hypothalamus, which indirectly affects the anterior pituitary gland's secretory function, reducing the contents of gonadotropins, estrogen, and progesterone, thereby causing follicle maturation inhibition and endometrial atrophy, leading to amenorrhea and changes in libido. On the other hand, antipsychotic drugs can affect the change curve of prolactin, and prolactin inhibits ovarian and pituitary gonadotropin, leading to a decrease in gonadotropin concentrations, leading to ovarian hypofunction and amenorrhea [10–15].

There were significant differences in estradiol, prolactin, and follicle-stimulating hormone between the progesterone and vitamin B6 groups after one month of treatment. The comparison of prolactin, uterine size and endometrial thickness is significantly different, and the vitamin B6 group is significantly lower than the progesterone group. The clinical treatment efficiency of vitamin B6 group is 95.00% significantly higher than the progesterone group 83.33%. There were no adverse reactions after medication in the progesterone and vitamin B6 groups. The results showed that the effect of progesterone combined with vitamin B6 in the treatment of antipsychotic amenorrhea was significantly better than that of progesterone alone, which could effectively improve the endocrine status of patients and provide a reference for the clinical treatment of antipsychotic amenorrhea. The endometrium undergoes significant changes due to the ovary secretion of estrogen and progesterone. Its physiological functions can be divided into the proliferative phase: It is equivalent to the follicular maturation phase, which is dominated by estrogen, and the endometrium is 1~5 mm. In the secretory phase, it is equivalent to the luteal phase and is dominated by progesterone. The presence of estrogen makes the endometrium continue to thicken, which is 6-10 mm. In the menstrual period, the endometrium is disintegrated and separated from the basal layer by the functional layer, which is the withdrawal of progesterone and estrogen. This study is conducted between the late proliferation and secretion period of the normal menstrual cycle, indicating that the endometrium has a certain degree of estrogen preparation. Still, because the patient takes antipsychotic drugs, the secretion of estrogen and progesterone is reduced, and the progesterone falls off. During bleeding, such patients are given progesterone treatment. There is withdrawal bleeding [16–20].

At the same time, female patients seriously impact their psychology due to amenorrhea, which can easily aggravate their depression and anxiety. In view of the problem of amenorrhea caused by antipsychotic drugs, it is necessary to solve the problem of hormonal abnormalities in patients. The combined treatment of progesterone and vitamin B6 can alleviate the phenomenon of irregular menstruation and amenorrhea [21–23]. Progesterone, also known as progesterone, is one of the progesterone secreted by the human ovaries. Progesterone can regulate the patient's hormone levels, protect the endometrium, promote the maturation and shedding of the endometrium, and restore the patient's menstrual cycle to normal [24–27]. Vitamin B is the catalyst of dopamine conversion, which can increase dopamine secretion in the patient's body. Dopamine and prolactin have a mutual inhibitory effect, thereby reducing the prolactin content and prompting the patient to resume the menstrual cycle [28, 29]. Therefore, the combined application of progesterone and vitamin B6 can adjust the hormone levels in patients with amenorrhea and promote the recovery of menstruation under the synergistic effect of the two [30–32]. The combination of progesterone and vitamin B in patients with amenorrhea caused by antipsychotic drugs can regulate the hormone secretion of patients, and the clinical application effect is better [33]. After 3 months of treatment, the patient's normal menstrual cycle was restored. At the same time, the above two drugs are safer, will not aggravate the patient's mental illness symptoms, and have no obvious adverse drug reactions [34]. Combined treatment of progesterone and vitamin B resulted in lower levels of prolactin, increased follicle stimulating hormone and estradiol, and normalized the menstrual cycle of patients [35].

Although this study also has shortcomings, vitamin B6 has a significant clinical effect on amenorrhea caused by antipsychotics, but the mechanism has not been studied in depth. The cases from the same hospital and were not representative of all situations. Subjective exclusion and inclusion may lead to biased results. To sum up, the effectiveness of progesterone combined with vitamin B6 in treating amenorrhea caused by antipsychotics is significantly better than simple progesterone, which can effectively improve the endocrine condition and provide a reference for clinical treatment of amenorrhea caused by antipsychotics.

## 5. Conclusion

Progesterone combined with vitamin B6 therapy can effectively improve the endocrine status of patients and provide a reference for the clinical treatment of antipsychotic amenorrhea.

## Figures and Tables

**Figure 1:** Research process.

**Table 1:** General information between the progesterone and vitamin B6 groups (*n*, $\bar{x}\pm \text{s}$).

Group	Average age (years)	Amenorrhea time (months)	Time of taking antipsychotic drugs (months)	Marital status	
				Unmarried	Married
Progesterone group (60)	29.78 ± 4.32	5 (3~6)	6.78 ± 2.32	23	37
Vitamin B6 group (60)	30.62 ± 2.66	4 (3~5)	6.62 ± 1.66	22	38
*χ* ^2^/*t*	− 1.283	0.121	0.434	0.036	
*P*	0.202	0.260	0.665	0.850	

**Table 2:** Endocrine indicators between the progesterone and vitamin B6 groups of patients ($\bar{x}\pm \text{s}$).

Group	Estradiol (pmol/L)		Prolactin (mU/L)		Follicle stimulating hormone (IU/L)	
	Before treatment	After 1 month of treatment	Before treatment	After 1 month of treatment	Before treatment	After 1 month of treatment
Progesterone group (60)	22.78 ± 4.32	64.74 ± 8.10	468.51 ± 27.32	412.78 ± 63.32	2.54 ± 0.33	4.67 ± 1.12
Vitamin B6 group (60)	22.62 ± 3.54	144.56 ± 9.14	472.55 ± 26.11	310.62 ± 52.22	2.46 ± 0.54	8.49 ± 2.17
*t*	0.222	-50.625	-0.828	9.641	0.979	-12.117
*P*	0.825	0.000	0.409	P <0.001	0.329	P <0.001

**Table 3:** Prolactin, uterine size and intima thickness between the progesterone and vitamin B6 groups ($\bar{x}\pm \text{s}$).

Group	Maximum diameter of uterus (cm)		Endometrial thickness (mm)		Prolactin (ͷg/L)	
	Before treatment	After 1 month of treatment	Before treatment	After 1 month of treatment	Before treatment	After 1 month of treatment
Progesterone group (60)	11.83 ± 1.20	11.64 ± 1.12	8.53 ± 1.27	6.20 ± 1.32	104.03 ± 15.32	25.15 ± 5.24
Vitamin B6 group (60)	11.79 ± 1.14	10.33 ± 0.71	8.44 ± 2.83	4.45 ± 0.81	105.62 ± 18.26	12.37 ± 2.37
*t*	0.187	7.652	0.225	8.753	− 0.517	17.213
*P*	0.852	*P* < 0.001	0.823	*P* < 0.001	0.606	*P* < 0.001

**Table 4:** Clinical efficacy between the progesterone and vitamin B6 groups (*n*(%)).

Group	Cure	Remarkable effect	Effective	Invalid	Efficiency
Progesterone group (60)	25 (41.67)	18 (30.00)	7 (11.67)	10 (16.67)	50 (83.33)
Vitamin B6 group (60)	27 (45.00)	16 (26.67)	14 (23.33)	3 (5.00)	57 (95.00)
*χ* ^2^					4.227
*P*					0.040

## Data Availability

No data were used to support this study.
